The article "Comparison of the sagittal profiles among thoracic idiopathic scoliosis patients with different Cobb angles and growth potentials" was retracted in 2015. Reason: compromised peer review.

# Comparison of the sagittal profiles among thoracic idiopathic scoliosis patients with different Cobb angles and growth potentials

**DOI:** 10.1186/1749-799X-9-19

**Published:** 2014-03-17

**Authors:** Bo Ran, Guo-you Zhang, Feng Shen, Jia-yu Chen, Ji-bin Wu, Feng-chao Zhao, Kai-jin Guo, Dun-yi Qi, Bing Zhou, Xiang-yang Chen, Xin-zhu Zhang, Yue-hua Qiao, Ming Li

**Affiliations:** 1 Department of Orthopedics, The Affiliated Hospital of Xuzhou Medical College, No. 99 Huaihai road, Xuzhou, Jiangsu 221006, China; 2 Department of Orthopedics, Changhai Hospital Affiliated to Second Military Medical University, Shanghai 200433, China; 3 Department of Orthopedics, Kunming General Hospital of Chengdu Military Command, Kunming 650032, China; 4 Department of Anesthesiology, The Affiliated Hospital of Xuzhou Medical College, No. 99 Huaihai road, Xuzhou, Jiangsu 221006, China; 5 Department of Otolaryngology, The Affiliated Hospital of Xuzhou Medical College, No. 99 Huaihai road, Xuzhou, Jiangsu 221006, China; 6 Institute of Audiology and Speech Science, The Affiliated Hospital of Xuzhou Medical College, Xuzhou, Jiangsu 221006, China

**Keywords:** Sagittal profiles, Idiopathic scoliosis, Thoracic kyphosis, Lumbar lordosis

## Abstract

**Background:**

Previous studies have demonstrated that pelvic incidence and sacral slope are significantly greater in idiopathic scoliosis patients compared with normal adolescents. However, whether these sagittal parameters are related to the progression of scoliosis remain unknown. The present was designed to determine the differences in the sagittal profiles among thoracic idiopathic scoliosis patients with different potentials for curve progression.

**Methods:**

Ninety-seven outpatient idiopathic scoliosis patients enrolled from June 2008 to June 2011 were divided to three groups according to different Cobb angles and growth potentials: (1) non-progression of thoracic curve group, Risser sign of 5 and Cobb’s angle < 40°; (2) moderate progression of thoracic curve group, Risser sign of 5 and Cobb’s angle ≥ 40°; and (3) severe progression of thoracic curve group, Risser sign ≤ 3 and Cobb’s angle ≥ 40°. All patients underwent whole spinal anteroposterior and lateral X-ray in standing position, and the sagittal parameters were measured, including thoracic kyphosis, lumbar lordosis, sacral slope, pelvic incidence, and pelvic tilt.

**Results:**

The average thoracic scoliosis Cobb’s angle in the non-progression group was significantly less than that in the moderate progression group (*P* < 0.01) and severe progression group (*P* < 0.01), but there was no statistical difference in the average thoracic scoliosis Cobb’s angle between the severe progression group and moderate progression group. The average thoracic kyphosis angle in the severe progression group (9° ± 4°) was significantly smaller than that in the non-progression group (18° ± 6°, *P* < 0.01) and moderate progression group (14° ± 5°, *P* < 0.05). No statistical differences were present in the average lumbar lordosis, sacral slope, pelvic incidence, and pelvic tilt among the three groups.

**Conclusions:**

Thoracic hypokyphosis is strongly related with the curve progression in thoracic idiopathic scoliosis patients, but not pelvic sagittal profiles.

## Introduction

Idiopathic scoliosis is the most common spinal deformity in human, affecting more than 2% of the adolescent population and resulting in more than 600, 000 physician visits annually [1]. Recent studies have discovered several risk factors associated with progression to a severe curve, including the delayed age of first menstruation [2], lower bone age [3], high Cobb’s angle at presentation [4], and decreased bone density [5]. In addition, some scholars report that there is a consistent loss of kyphosis in thoracic scoliosis patients compared with normal control or patients with thoracolumbar curves [6,7] and scoliosis progresses faster in patients with minor thoracic kyphosis [8]. Pelvic incidence and sacral slope are also shown to be significantly greater in idiopathic scoliosis patients compared with normal adolescents [7]. However, whether these sagittal parameters are related to the progression of scoliosis remain unknown. In this study, we aimed to compare the sagittal profiles among the thoracic idiopathic scoliosis patients with three different progression potentials.

## Methods

### Patients

A total of 97 right thoracic curve idiopathic scoliosis patients were admitted to our hospital from June 2008 to June 2011. No treatment was adopted before the visit to interfere the nature history of the scoliosis progression in all 97 enrolled patients. All human studies have been approved by the hospital ethics committee and performed in accordance with the ethical standards. Written informed consent was obtained from all the participants or their parents.

All of these 97 patients underwent clinical and radiological examinations by expert spinal surgeons and were divided to three groups according to the different progression potentials: (1) non-progression of thoracic curve group, Risser sign of 5 and Cobb’s angle < 40°; (2) moderate progression of thoracic curve group, Risser sign of 5 and Cobb’s angle ≥ 40°; and (3) severe progression of thoracic curve group, Risser sign ≤ 3 and Cobb’s angle ≥ 40° [9].

### Imaging measurement index

All of these 97 patients underwent whole spinal anteroposterior and lateral X-ray in standing position. The X-ray imaging was inputted into the computer and digitally analyzed with image-pro plus 6.0 software [10] to obtain the following sagittal parameters: (1) thoracic kyphosis, the Cobb’s angle between the cranial superior endplate of T5 and the caudal inferior endplate of T12 (positive values are defined as kyphosis, while negative values are defined as lordosis); (2) lumbar lordosis, the Cobb’s angle between the cranial superior endplate of L1 and the caudal superior endplate of S1 (positive values are defined as lordosis, while negative values are defined as kyphosis); (3) sacral slope, the angle between the upper end plate of S1 and the horizontal line; (4) pelvic incidence, defined as the angle between the perpendicular of the upper endplate of S1 and the line joining the middle of the upper endplate of S1 and the hip axis (midway between the centers of the two femoral heads); and (5) pelvic tilt, the angle between the vertical line and the line joining the middle of the upper endplate of S1 and the hip axis (positive when the hip axis lies in front of the middle of the upper endplate of S1). None of the patients underwent treatment during study.

### Statistical analysis

All data were analyzed by SPSS 13.0 software package (SPSS Inc., Chicago, IL, USA) and expressed as mean ± standard deviation (SD). The difference between three groups was analyzed by one-way analysis of variance (ANOVA). *P* < 0.05 was considered statistically significant.

## Results

### General data

The general characteristics of these three groups are shown in Table 1. Thirty-one patients were assigned into the non-progression group, in which 29 patients were female and 2 patients were male; the average age was 17.9 years old (14–24 years old), and the average thoracic Cobb’s angle was 30° ± 6°. Thirty-four patients belonged to the moderate progression group, in which 32 patients were female and 2 patients were male, the average age was 18.7 years old (16–25 years old), and the average thoracic Cobb’s angle was 50° ± 8°. Thirty-two patients were categorized into the severe progression group, in which 29 patients were female and 3 patients were male, the average age was 13.8 years old (11–16 years old), and the average thoracic Cobb’s angle was 51° ± 7°. There was no statistical difference among these patients in sex ratio. But there were significant differences in average age, average thoracic Cobb’s angle, and average Risser sign among the three groups. The average age in the severe progression group was significantly less than that in the non-progression group (*P* < 0.01) and the moderate progression group (*P* < 0.01), while there was no statistical difference in the average age between the non-progression group and the moderate progression group (*P* = 0.761). The average thoracic Cobb’s angle in the non-progression group was significantly smaller than that in the moderate progression group (*P* < 0.01) and the severe progression group (P < 0.01), but no statistical difference in the average thoracic Cobb’s angle was observed between the severe progression group and the moderate progression group (*P* = 0.622). The Risser sign of the non-progression group and the moderate progression group was 5°. But the average Risser sign of the severe progression group was 1.8 which was significantly less than that in the moderate progression group (*P* < 0.01) and the non-progression group (*P* < 0.01).

**Table 1:** General data of idiopathic scoliosis patients with non-progression, moderate progression, and severe progression of thoracic curve

**Group**	**Cases**	**Age (years)**	**Gender (male/female)**	**Thoracic Cobb’s (°)**	**Risser sign**
Non-progression	31	17.9 ± 2.1	2/29	30 ± 6^ab^	5
Moderate progression	34	18.7 ± 2.4	2/32	50 ± 8	5
Severe progression	32	13.8 ± 1.3^a^	2/29	51 ± 7	0–3 (average 1.8)^a^

^a^*P* < 0.01, compared to the moderate progression group; ^b^*P* < 0.01, compared to the severe progression group.

The typical cases in each group are shown in Figures 1,2,3.

**Figure 1:** **An 18-year-old female thoracic idiopathic scoliosis patient.** Risser sign was 5. The thoracic scoliosis Cobb’s angle was 30°, and the thoracic kyphosis Cobb’s angle was 28°. **(A)** The whole spinal anteroposterior in standing position. **(B)** Lateral X-ray in standing position.

**Figure 2:** **A 16-year-old female thoracic idiopathic scoliosis patient.** Risser sign was 5. The thoracic scoliosis Cobb’s angle was 42°, and the thoracic kyphosis Cobb’s angle was 15°. **(A)** The whole spinal anteroposterior in standing position. **(B)** Lateral X-ray in standing position.

**Figure 3:** **A 15-year-old female thoracic idiopathic scoliosis patient.** Risser sign was 3. The thoracic scoliosis Cobb’s angle was 50°, and the thoracic kyphosis Cobb’s angle was 7°. **(A)** The whole spinal anteroposterior in standing position. **(B)** Lateral X-ray in standing position.

### Comparison of the sagittal parameters

The sagittal parameters of these three groups are displayed in Table 2. The average thoracic kyphosis angle was 18° ± 6°, 14° ± 5°, and 9° ± 4° in the non-progression group, moderate progression group, and the severe progression group, respectively. Statistical analysis indicated that the average thoracic kyphosis angle in the severe progression group was significantly smaller than that in the non-progression group (*P* < 0.01) and moderate progression group (*P* < 0.05). The average thoracic kyphosis angle in the moderate progression group was also significantly smaller than that in the non-progression group (*P* < 0.01). No statistical differences were present in the average lumbar lordosis, sacral slope, pelvic incidence, and pelvic tilt between the above three groups (*P* > 0.05).

**Table 2:** Sagittal parameters of idiopathic scoliosis patients with non-progression, moderate progression, and severe progression of thoracic curve (°, X ± S)

**Group**	**Thoracic kyphosis angle**	**Lumbar lordosis Cobb’s angle**	**Sacral slope Cobb’s angle**	**Pelvic incidence Cobb’s angle**	**Pelvic tilt angle**
Non-progression	18 ± 6	51 ± 7	35 ± 6	42 ± 9	8 ± 6
Moderate progression	14 ± 5^a^	46 ± 9	36 ± 7	45 ± 11	9 ± 7
Severe progression	9 ± 4^ab^	50 ± 8	38 ± 6	46 ± 9	8 ± 7

^a^*P* < 0.01, compared to the non-progression group; ^b^*P* < 0.05, compared to the moderate progression group.

## Discussion

It is reported that idiopathic scoliosis deformity progresses until skeletal maturity. Skeletal maturity was defined as the Risser sign of 4 or 5 [4]. In addition, the scoliosis of a Cobb angle greater than 40° has been reported to have 70% progression rate after skeletal maturity, whereas those less than 30° have little progression [11]. Thus, in this study, we defined the curve progression according to the Risser sign and Cobb angle [9]. The grouping method in our study may reflect truly the three different scoliosis progressions. The Risser sign of the non-progression patients and the moderate progression patients reached to 5 in our study, indicating the growth potential is very small and the scoliosis progression tends towards stability. But the average Cobb’s angle of the moderate progression patients was greater obviously than that of the non-progression patients, so the scoliosis progression in the moderate progression patients was greater than that in the non-progression patients. The average Cobb’s angle of the moderate progression patients was the same as that of the severe progression patients, but the Risser sign of the severe progression patients was below 3 (the average Risser sign was only 1.8), so the growth potential of the severe progression patients was great and the scoliosis progression continued. Thus, the scoliosis progression in the severe progression patients was still greater than that in the moderate progression patients.

Although the etiology is complex, progressive adolescent idiopathic scoliosis is generally attributed to relative anterior spinal overgrowth from a mechanical mechanism during the adolescent growth spurt, which leads to thoracic hypokyphosis followed by increasing axial rotational instability [12,13]. This theory is further confirmed by some clinic studies. For example, Rigo et al. found that the patients with more severe thoracic curves had smaller thoracic kyphotic angles [14]. Ylikoski reported the sagittal profiles of 535 adolescent idiopathic scoliosis patients and found that the mean progression velocity of major curves was 2.8° every year in the patients with minor thoracic kyphosis, while 1.8° every year in the patients with greater thoracic kyphosis [8]. Our results were also consistent with the above observation, showing that the average thoracic kyphosis angle in the severe progression group was significantly smaller than that in the non-progression group and the moderate progression group significantly.

Interestingly, thoracic hypokyphosis is only observed in the thoracic scoliosis patients, and there is no significant difference in the thoracic kyphosis between the lumbar scoliosis patients and normal people [7]. These suggest that the pathogenesis of the thoracic idiopathic scoliosis patients may be different from that in the lumbar idiopathic scoliosis patients, and the relationship between the thoracic hypokyphosis and the scoliosis progression seems to be more evident in the thoracic idiopathic scoliosis. Thus, only the thoracic idiopathic scoliosis patients were selected as the study objects, which make our analysis more scientific and targeted. In addition, the included patients had no history of any treatments before, which can prevent the scoliosis’ natural progression from disturbance.

Other than thoracic kyphosis, we also evaluated the relationship between other sagittal parameters and scoliosis progression, including lumbar lordosis, sacral slope, the pelvic incidence, and the pelvic tilt. Pelvic incidence and pelvic tilt are describing pelvic rotation around the center of femoral head (hip axis). This rotation represents a pelvic compensatory mechanism in response to the change in the spinal alignment. Some scholars found that the pelvic incidence in the idiopathic scoliosis patients was greater than the normal people, so they thought that an increase in pelvic incidence was one of the scoliosis progressive factors [7]. Some papers reported that pelvic incidence had a strong correlation with lumbar scoliosis at sagittal plane in both scoliosis patients and normal subjects [15,16], which indirectly demonstrates that lumbar scoliosis may have an effect on the sagittal balance. However, in our study, there was no statistical difference about the sacral slope, pelvic incidence, and pelvic tilt angle between the above three groups, indicating that there may be no relationship between the pelvic profile and the thoracic progression.

## Conclusion

The results of this study support that thoracic hypokyphosis is strongly related with the curve progression in thoracic idiopathic scoliosis patients, but not pelvic sagittal profiles.

## Competing interests

The authors declare that they have no competing interests.

## Authors’ contributions

BR, GYZ, and FS participated in the design of this study and performed the statistical analysis. JYC, JBW, and FCZ carried out the study, together with KJG, collected important background information, and drafted the manuscript. DYQ, BZ, XYC, XZZ, YHQ, JHG and ML conceived of this study and participated in the design and helped to draft the manuscript. All authors read and approved the final manuscript.

## Authors’ information

Bo Ran is the first author,Guoyou Zhang and Feng Shen are co-first authors Xiangyang Chen is the corresponding author, Junhui Guan and Kaijin Guo are co-corresponding authors.
